The article "Mechanical stimulation induced osteogenic differentiation of BMSCs through TWIST/E2A/p21 axis" was published in 2020. Journal: Biosci Rep.

# Mechanical stimulation induced osteogenic differentiation of BMSCs through TWIST/E2A/p21 axis

**DOI:** 10.1042/BSR20193876

**Published:** 2020-05-04

**Authors:** Qingyuan Guo, Ying Liu, Renhao Sun, Fang Yang, Pengyan Qiao, Rong Zhang, Ling Song, Lingling E, Hongchen Liu

**Affiliations:** 1 Institute of Stomatology, Chinese PLA General Hospital, Beijing 100853, China; 2 Department of Stomatology, Qingdao Municipal Hospital Group, Qingdao University, Qingdao, Shandong 266011, China

**Keywords:** BMSCs, mechanical stimulation, osteogenic differentiation, p21

## Abstract

The relationship between mechanical force and alveolar bone remodeling is an important issue in orthodontics because tooth movement is dependent on the response of bone tissue to the mechanical force induced by the appliances used. Mechanical cyclical stretch plays an essential role in the cell osteogenic differentiation involved in bone remodeling. However, the underlying mechanisms are unclear, particularly the molecular pathways regulated by mechanical stimulation. In the present study, we reported a dynamic change of p21 level in response to mechanical cyclical stretch, and shRNA-p21 in bone marrow mesenchymal stem cells (BMSCs) induced osteogenic differentiation. The mechanism was mediated through TWIST/E2A/p21 axis. These results supported the mechanical stimulation-induced osteogenic differentiation is negatively regulated by p21.

## Introduction

The biological basis of orthodontic tooth movement is bone [1,2], and there are many factors affecting alveolar bone remodeling [3]. Mechanical force is one of the most important factors [4]. Bone marrow mesenchymal stem cells (BMSCs) are proliferated and differentiated by mechanical stimulation, which is important for orthodontic tooth movement and orthodontic maintenance [5]. Because bone marrow, the original environment of BMSCs, is hypoxic with the oxygen tension approximately 1–7% [6], we hypothesized that hypoxic microenvironment provides more benefits than normoxia. Our previous study provided evidence that cyclic stretch activated the hypoxic culture environment of BMSCs, and initiated the HIF-TWIST pathway [7]. Also, mechanical tension stimulated osteogenic differentiation of BMSCs [8], and the differentiation is different when the loading condition is different [9]. However, it has not yet been elucidated that the mechanism among mechanical stimulation, HIF-TWIST axis and osteogenic differentiation of BMSCs.

Hypoxia has been known to regulate several cellular processes and signal transductions via the expression of hypoxia inducible factor-1 (HIF-1), a heterodimer consisting of the constitutively expressed aryl hydrocarbon receptor nuclear translocator (ARNT) and the hypoxic response factor HIF-1α [10]. HIF-1α is regulated by the cellular O_2_ concentration and determines the transcriptional activity of HIF-1 [11]. TWIST, a basic helix–loop–helix (bHLH) transcription factor, promotes tumor metastasis by inducing epithelial–mesenchymal transition (EMT) [12]. Recently, the HIF-TWIST axis has been demonstrated in head and neck cancer [13] and follicular thyroid cancer [14]. Stem cells and cancer cells share a lot of similarities in gene expression, cellular processes and signal transductions, but there are not many studies researching the effects of HIF-TWIST on normal stem cells. Recent studies have shown that E2A and TWIST both belong to the bHLH protein family [15]. E2A can activate the expression of cyclin-dependent kinases (CDKs) inhibitor p21 gene [16,17]; p21 also plays an important role in the differentiation of osteoblasts and myoblasts [18,19]. Although E2A-p21 expression and senescence have been reported to impair the efficiency of somatic cell reprogramming [20,21], the roles of E2A-p21 in regulating pluripotency and stem cell properties of BMSCs have not been elucidated.

The article "Mechanical stimulation induced osteogenic differentiation of BMSCs through TWIST/E2A/p21 axis" was published in 2020. Journal: Biosci Rep.

In the present study, we have found that mechanical stimulation not only induced osteogenic differentiation of BMSCs, but also affected the expression of TWIST and E2A-p21. During mechanical osteo-induction of BMSCs, TWIST and E2A-p21 were not only simply linearly regulated, but p21 also negatively regulated the expression of TWIST and E2A. The underlying mechanism mediating the increase in BMSCs osteogenic differentiation by mechanical stimulation is through down-regulation of TWIST/E2A/p21 axis.

## Materials and methods

### Isolation and identification of BMSCs

The experiments took place at Qingdao Municipal Hospital, and the study design was submitted to and approved by the Qingdao Municipal Hospital Medical Ethics Committee (No. 2019035). Sprague–Dawley rats (140 ± 10 g, 4-week-old male) were treated in painless state by anesthesia combined with nasal inhalation of ether and intraperitoneal injection of pentobarbital sodium, breaking the neck to death (Qingdao Municipal Hospital Experimental Animal Center, Qingdao, China). BMSCs primary cell culturing was carried out as described previously with minor modification [22]. The tibias and femurs were isolated from the rats. Under aseptic circumstances, the bone marrow was flushed out and mixed with complete α minimal essential medium (α MEM; HyClone, Thermo, U.S.A.) supplemented with 15% fetal bovine serum (FBS, Gibco, U.S.A.), 100 U/ml penicillin and 100 μg/ml streptomycin. The harvests were plated into a culture flask, and were incubated for 3 days in a humidified atmosphere containing 5% CO_2_ at 37°C to allow attachment of adherent cells. Culturing medium was changed every 3 days to remove the non-adherent cells and to provide nutrition that the cells needed.

The article "Mechanical stimulation induced osteogenic differentiation of BMSCs through TWIST/E2A/p21 axis" was published in 2020. Journal: Biosci Rep.

### Flow cytometric characterization of BMSCs

The expression of mesenchymal and non-mesenchymal stem cell-associated surface markers that are the characters of the immunophenotype of BMSCs were measured by flow cytometric analysis at early passages (P3). Briefly, approximately 5 × 10^5^ liberated adherent BMSCs were detached from the culture flasks and suspended in PBS containing 3% FBS in different EP tubes, and the following antibodies were incubated for 20 min at room temperature in the dark: CD4, CD44, CD45, CD90, CD105 (eBioscience, U.S.A.). A negative panel of the following surface antigens was incubated simultaneously as a group in the same sample. Cell suspension without antibodies served as a control group to determine background fluorescence. After 1 h, the cells were washed with PBS containing 3% FBS for three times and 300 ml of the suspension was added into the testing tubes, equipped with laser emission at 488, 633 and 407 nm. The FITC and PE channels were used to detect the emission of conjugated surface antigens [23]. Finally, the samples were measured by flow cytometric analysis using a Beckman Coulter Epics XL cytometer (Beckman Coulter, Fullerton, CA, U.S.A.).

### Mechanical cyclic stretch load application

BMSCs were plated at a density of 1 × 10^5^ cells/ml in 2 ml medium on six-well flexible silicone rubber BioFlex™ plates coated with rat tail collagen type I (Flexcell International Corp., Hillsborough, NC, U.S.A.). The cells were cultured for 48 h to allow them to attach and reach 80–90% confluence, at which time the growth medium was replaced, and mechanical stimulation was applied. A cyclic mechanical stretch with a 1 Hz sinusoidal curve set at 5% elongation was applied for each treatment respectively, using FX 5000T™ Flexcell Tension Plus™ unit (Flexcell International Corp.). The cultures were incubated in a humidified atmosphere at 37°C and 5% CO_2_ while stretching [24]. The BMSCs were collected after 0, 3, 6, 9 and 12 h of stretch stimulation.

### RNA interference of p21 in BMSCs

The GFP, dominant-negative form of BMSCs (p21-shRNA) and wild-type BMSCs (WT) were cloned into a lentiviral vector pGMLV-SC1 purchased from Genomeditech (Shanghai, China). Lenvirius was packaged and amplified in HEK293 cells. Specific gene silencing was achieved by transfection of double-stranded small interfering (si) RNA targeting Rat p21 (Gene ID: 24525) consisting of 5′-GGAGTTATGGGATTCCATTCA-3′. The scrambled small RNA (5′-TTCTCCGAACGTGTCACGT-3′) was also confirmed as non-silencing double-stranded RNA and used as a control in the current study (NC). In these experiments, all the three groups of cells had a GFP-tagged internal ribosome entry site for monitoring infection efficiency. p21-shRNA and NC cells were infected at a multiplicity of infection (MOI) of 10, unless otherwise noted. At this dose, 48–72 h after infection, most of the cells were GFP positive, and both the p21-shRNA and NC cells were well expressed. Transfection of or cDNA was performed by using the siLentFect Lipid Reagent (Bio-Rad) according to instructions from the manufacturer [25]. The efficiency of p21silencing was assessed by Western blot and real-time PCR analysis. The p21 antibody was purchased from Abcam (U.S.A.).

The article "Mechanical stimulation induced osteogenic differentiation of BMSCs through TWIST/E2A/p21 axis" was published in 2020. Journal: Biosci Rep.

### Quantitative real time RT-PCR

Total RNA was isolated by using RNAiso Plus (Takara, Japan), following the manufacturer’s instructions [26]. Concentration of the isolated RNA was determined at 260 nm with using Gene Quant Pro (Amersham Biosciences, U.S.A.) and reverse transcription was performed with Prime Script® RT reagent Kit With gDNA Eraser (Takara, Japan). Quantitative PCR was performed by using SYBR®Premix Ex Taq™ (Takara, Japan) according to the manufacturer’s instructions [26]. The conditions of the quantitative real time RT-PCR (qPCR) were as follows: denaturation at 95°C for 30 s, 40 cycles at 95°C for 50 s and 60°C for 20 s and a final dissociation stage (65°C for 15 s) was added at the end of the amplification procedure. GAPDH was used as an internal control. The data were analyzed using comparative *C*_t_ (2^−ΔΔ*C*_t_^) method and expressed as a fold change respective to the control. Each sample was analyzed in triplicate. The primer sequences used in the present study are listed in Table 1.

**Table 1:** Oligodeoxynucleotide primers used for qPCR

Name	Sequence	Length (bp)
GAPDH-F	CATTCTTCCACCTTTGAT	92
GAPDH-R	CTGTAGCCATATTCATTGT	
TWIST-F	AGATTCAGACCCTCAAACT	88
TWIST-R	CTTGCCATCTTGGAGTCC	
E2A-F	GAACCAGTCTCAGAGAAT	77
E2A-R	GGAACATCATACTGAAGTC	
p21-F	GATGTCCGACCTGTTCCA	75
p21-R	GCTCAACTGCTCACTGTC	
RUNX2-F	AATGCCTCTGCTGTTATG	109
RUNX2-R	TTGTGAAGACCGTTATGG	
BMP2-F	CATCACGAAGAAGCCATC	92
BMP2-R	TCATCAGTAGGGACAGAAC	
OSTERIX -F	CGGGACTCAACAACTCTG	75
OSTERIX -R	TTTGGAGGCTGAAAGGTC	

### Western blotting analysis

Cell–aggregate lysates were extracted by lysing the cells in by Western and IP protein extraction reagent (Beyotime, China) with a protease inhibitor cocktail (Sigma, U.S.A.) for 5 min on ice, and then the concentration of total protein was determined with BCA protein assay (Keygen Biotech, China) following the manufacturer’s recommended protocol [27]. After being heated for 5 min at 100°C in a loading buffer, loaded 20 mg of each detected protein sample was separated by sodium dodecyl sulfate/polyacrylamide gel electrophoresis (SDS/PAGE) and then was electro-transferred into polyvinylidenedifluoride (PVDF) membranes (Millipore, Billerica, MA, U.S.A.). Then the PVDF membranes were blocked for 0.5 h with TBS containing 5% non-fat dry milk powder and 0.05% Tween 20 and then incubated overnight at 4°C with the primary antibodies against p21, TWIST, RUNX2, BMP2, E2A, OSTERIX and GAPDH (Abcam, U.S.A.). The membranes were washed three times for 10 min each with TBS containing 0.05% Tween 20. Bound primary antibodies were detected by incubating for 1 h with horseradish peroxidase–conjugated goat anti-mouse or anti-rabbit IgG (CWBio, China). The membranes was washed and developed using a ECL Reagent (Millipore, U.S.A.) following the manufacturer’s recommended protocol [27], and were quantified using the Image-Quant software.

The article "Mechanical stimulation induced osteogenic differentiation of BMSCs through TWIST/E2A/p21 axis" was published in 2020. Journal: Biosci Rep.

### Statistical analysis

All data were presented as mean ± SD and statistical significance was evaluated by analysis of variance using SPSS software (IBM, Armonk, U.S.A.). The statistical significance was considered at *P*<0.05.

## Results

### Identification of isolated BMSCs

After adherent culture and subculture *in vitro*, the cell growth is gradually stable, and the cell morphology is uniform and long fusiform. The BMSCs passed to the 7th day appeared a uniform density distribution and fibroblast-like morphology. The results of flow cytometry showed that the cell surface antigens CD44, CD90 and CD105 were positive, while the CD4 and CD45 results were negative. The above results were consistent with the surface-specific antigen of BMSCs (Figure 1).

**Figure 1:** Identification of isolated BMSCs (**A**) BMSCs exhibited a uniform colony on the 3rd day, a flattened, elongated shape on the 5th day, a high density and fibroblastic-like morphology on the 7th day (magnification, 100×). (**B**) Flow cytometric analysis of antigen expression of BMSCs showed the percentages of positive cells are 95.6% (CD44), 92.7% (CD90), 97.5% (CD105), 4.75% (CD4), 4.14% (CD45), respectively.

### Mechanical stimulation induced osteogenic differentiation and p21 expression of BMSCs

Mechanical stimulation was applied to BMSCs and the progress of osteogenesis was examined. The quantitative data analysis of RUNX2 (**P<0.01) and BMP2 (**P<0.01) indicated an increased tendency after stimulated by 1 Hz, 5% stretch loading for 0, 3, 6, 9, 12 h. TWIST (*P<0.05) and p21 (**P<0.01) also presented a time-dependent rise, while mRNA and protein expression of transcription factor E2A (***P<0.001) reduced subjected to cycling stretch (Figure 2). It is indicated that cyclic stretch can promote osteogenic differentiation of BMSCs and affect the expression of transcription factors.

The article "Mechanical stimulation induced osteogenic differentiation of BMSCs through TWIST/E2A/p21 axis" was published in 2020. Journal: Biosci Rep.

**Figure 2:** Mechanical stimulation induced osteogenic differentiation and p21 expression of BMSCs (**A**) The quantitative data analysis of BMP2, RUNX2, TWIST and p21 indicated an increased tendency, while E2A decreased after stimulated by the 5% stretch exhibited for 0, 3, 6, 9 and 12 h (*P<0.05, **P<0.01, ***P<0.001). (**B**) Protein expression by Western blotting showed the same trend, and GAPDH was used as a loading control.

### Identification of BMSCs with RNA interference of p21

BMSCs without any treatment (WT), with RNA interference of p21 (p21-shRNA) and non-silencing double-stranded RNA (NC, used as control) were observed under fluorescence microscope. After alignment, the fragment sequence inserted in the recombinant lentivirus was identical to the designed oligo sequence, and the p21 RNA interference lentiviral vector was successfully constructed. The virus titer was 5 × 10^8^ TU/ml. Compared with the WT group and the NC group, the proportion of p21-shRNA BMSCs in the S phase and G_1_+S phase were significantly increased, while the cells in the G_1_ and G_2_ phases were decreased. Down-regulation of the p21 gene caused a significant reduction in p21 mRNA (**P<0.01) and protein compared with the WT and NC groups (Figure 3).

**Figure 3:** Identification of BMSCs with RNA interference of p21 (**A**) Immunofluorescence microscopy observations at 96 h after lentivirus-transfected 293T (×100). Cells of p21-shRNA and NC groups were both green. (**B**) Flow cytometry to detect cell cycle. (**C**) mRNA and protein expression of p21 in three groups. (***P<0.001).

### p21-shRNA BMSCs increased osteogenic difference induced by mechanical cycling stretch

After loading the cells of WT, p21-shRNA and NC groups with cyclic stretch of 1 Hz, 5% and 9 h, the results of qPCR showed that TWIST (**P<0.01) was inhibited, and E2A (***P<0.001) was greatly promoted; mRNA expression of osteogenic factors RUNX2 (**P<0.01) and OSTERIX (***P<0.001) was detected after down-regulating p21. There was a decreasing trend in BMP2 (*P<0.05) with the absence of p21. Western blotting showed that protein results for the above factors are consistent with the trend of qPCR (Figure 4).

**Figure 4:** p21-shRNA BMSCs increased osteogenic difference induced by cycling stretch (**A**) Expression of TWIST, p21, BMP2, E2A, OSTERIX and RUNX2 mRNA affected by 5%, 1 Hz cycling stretch for 9 h in three groups. The values are the mean ± standard deviation (*P<0.05, **P<0.01, ***P<0.001). (**B**) Expression of TWIST, p21, BMP2, E2A, OSTERIX and RUNX2 analyzed by Western blotting after 5%, 1 Hz cycling stretch for 9 h in three groups. GAPDH was used as a loading control.

The article "Mechanical stimulation induced osteogenic differentiation of BMSCs through TWIST/E2A/p21 axis" was published in 2020. Journal: Biosci Rep.

## Discussion

In the current study, we have shown that the p21 expression and production was affected by the mechanical stimulation. In addition, knockdown of p21 induced BMSCs osteogenic differentiation and increased stem cell pluripotency subjected to mechanical cycling stretch. We further proved the bone remodeling could be activated under cyclic stretch, such as those of the bone marrow hypoxic microenvironment, by a signaling pathway involving the suppression of TWIST/E2A/p21 axis. The E2A-p21 pathway plays an important role in cell-cycle arrest involved in differentiation of various cell types [17]. Previously, osteogenic differentiation of osteoblastic cell lines was found to be closely associated with the mechanical stimulation [28,29]. To our knowledge; this is the first paper demonstrating the regulation of normal stem cell properties by TWIST via direct regulation of E2A-p21 pathway. This suggested that in the process of osteogenesis, osteogenic differentiation is continuously enhanced by appropriate mechanical stretch. In addition, the osteogenesis process simultaneously negatively regulated via the TWIST/E2A/p21 axis. Studies have shown that p21 protein participates in many cell responses, inhibits cell proliferation, promotes cell differentiation and accelerates cell aging [30–32]. In addition, p21 also plays an essential role in the biological behavior of BMSCs [33–35]. The expression of p21 in BMSCs cultured *in vitro* increased with the passage times. More importantly, it was found that decreased expression of p21 could improve bone repair ability in rodent skull defect models [36]. We found that after p21 was suppressed by RNA interference technology, the total S phase of cells in p21-shRNA group increased significantly, which is much higher than WT group and NC group [37].

In this experiment, we found that down-regulating p21 promoted the expression of E2A and inhibited the expression of TWIST by mechanical cyclic tension. It can be found that p21, as a downstream gene of TWIST and E2A, regulates the expression of TWIST by positive feedback and E2A by negative feedback. Research showed that E2A and TWIST could compete with Snail to bind E-box to control the expression of p21WAF/Cip1 and regulate the proliferation and differentiation of osteoblasts [38]. TWIST can also inhibit the expression of p21 by binding to E2-box and E5-box, increase the osteogenic potential of stem cells and maintain the characteristics of senile stem cells [39]. Therefore, we speculated that the transcriptional level of p21 decreased after silencing p21 under the stimulation of cyclic stretch. Failure to bind E2A specifically to p21 promoter resulted in accumulation of E2A, whereas increased binding of E2A to TWIST resulted in decreased expression of TWIST.

The article "Mechanical stimulation induced osteogenic differentiation of BMSCs through TWIST/E2A/p21 axis" was published in 2020. Journal: Biosci Rep.

Further review of the literature shows that transcription factor TWIST is a downstream gene of HIF-1α [40]. TWIST and HIF-1α inhibit the differentiation of MSC into osteocytes through direct or indirect interaction with RUNX2. TWIST can inhibit the expression of RUNX2 in BMSCs and the down-regulation other osteogenic marker. [39]. RUNX2 is the most specific gene in the process of osteogenesis, which is relatively early expressed in the osteogenic differentiation of MSCs [41]. OSTERIX is a downstream gene of RUNX2, also an essential transcription factor in osteogenic differentiation. RUNX2 and osterix are both considered as markers of early osteogenic differentiation [42]. OSTERIX is necessary to guide mesenchymal stem cells to osteoblasts and induce bone formation [43]. We found that cyclic tension can promote the expression of RUNX2 and OSTERIX in BMSCs, and p21 protein was involved in the regulation of osteogenic differentiation. However, p21 had different regulatory effects on RUNX2, OSTERIX and BMP2. Down-regulating p21 increased the expression of RUNX2 and OSTERIX, but decreased BMP2 to some extent. We speculated that p21 may play an important role in the regulation of osteogenic differentiation induced by mechanical cyclic stretch. It can not only be promoted by mechanical stimulation, but also maintain the relative balance between the osteogenic factors.

## Conclusion

In conclusion, we demonstrate that mechanical cycling strain can promote TWIST and inhibit E2A. TWIST and E2A interact in some way and activate the expression of p21. Down-regulating p21 could enhance the osteogenic differentiation. The results suggest that p21 plays an essential role in osteogenic differentiation induced by mechanical stimulation, and the mechanism was mediated through TWIST/E2A/p21 axis (Figure 5).

**Figure 5:** Schematic diagram of the mechanism through E2A-p21 by HIF-TWIST axis in regulating osteogenic differentiation of BMSCs under mechanical stimulation

## Abbreviations

bHLH: basic helix–loop–helix
BMSC: bone marrow mesenchymal stem cell
FBS: fetal bovine serum
HIF-1: hypoxia inducible factor-1
PVDF: polyvinylidenedifluoride
qPCR: quantitative real time RT-PCR
